# Research on Application of Data Mining Algorithm in Cardiac Medical Diagnosis System

**DOI:** 10.1155/2022/7262010

**Published:** 2022-05-14

**Authors:** Jianyong Peng, Xinhao Zhang, Lina Wang, Fang Zhu, Nana Zhou, Yansong Zuo, Tao Zhou, Yuan Gao

**Affiliations:** ^1^Ultrasonography Department, Rizhao International Heart Hospital, Rizhao, 276825, China; ^2^Department of Critical Care Medicine, Rizhao International Heart Hospital, Rizhao, 276825, China; ^3^Rizhao Hospital Affiliated to Qingdao University Rizhao International Heart Hospital, Rizhao, 276825, China; ^4^Rizhao Hospital Affiliated to Qingdao University, Rizhao, 276825, China; ^5^Cardiac Surgery, Rizhao International Heart Hospital, Rizhao, 276825, China; ^6^Oral and Maxillofacial Surgery, Rizhao Stomatological Hospital, Rizhao, 276825, China

## Abstract

Heart disease is a very common high-incidence disease. Due to the wide variety of pathology of heart disease, how to improve the medical diagnosis of heart disease and carry out earlier intervention and treatment is a problem that needs to be solved urgently. The paper adds the decision tree algorithm and its comparison and proposes an optimized classification algorithm Co-SVM. Based on the establishment of a heart disease diagnosis classifier based on data mining algorithms, it is aimed at exploring which of these four algorithms is more suitable for heart disease diagnosis problems and optimizing them. A brief description of the cause, influencing factors, and acquired data of heart disease can be seen from the accuracy and scientificity of the data, which further enhances the authenticity and reliability of the clinical diagnosis model of heart disease. At the same time, the ultrasound diagnosis technology of heart disease is introduced, and the important role of ultrasound diagnosis technology in the medical diagnosis of heart disease is discussed. This thesis uses the heart disease clinical data set to establish a heart disease diagnosis classifier based on the decision tree algorithm, neural network algorithm, support vector machine algorithm, and Co-SVM algorithm. Through experimental comparison and analysis, the optimal classification is selected according to the obtained results. The algorithm is Co-SVM algorithm. The experimental results show that the proposed Co-SVM algorithm has a higher accuracy rate than the other three classic algorithms, and the effectiveness of the Co-SVM algorithm is verified by the evaluation results of multiple algorithms. By applying the Co-SVM algorithm in the medical diagnosis system, it is helpful to assist doctors in making more accurate and precise diagnosis of the condition.

## 1. Introduction

Today, with the continuous improvement of the economic level, people's living standards are also constantly improving, and people's attention to life has also changed [1, 2]. Most people “free themselves” from the first concern about food and clothing. Pay more attention to spiritual richness. With the continuous development and change of economy and society, people's living and working environment is getting worse and worse. Terms that have never appeared before, such as air pollution, fog, car exhaust, and waste oil, are slowly beginning to invade people's lives and bring harm to people's bodies [3–5]. At the same time, as the pace of society accelerates, people have begun to receive pressure from all aspects, competition in study, life, and work. What followed was that their physical condition was much worse than before, and many people's bodies began to be in a “subhealthy” state. In this context, people began to pay more attention to health-related issues, paying attention to their own health while also paying attention to the health of others. People gradually agree that people should be treated immediately when a disease occurs, and doctors should also make a good diagnosis or accurate prediction and prevention of the disease, to better reduce the patient's pain and achieve accurate prediction, diagnosis, and treatment [6].

Since 1990s, heart disease and cardiovascular disease have been the main causes of death in our country. Judging from the reports of the Chinese Society of Cardiology over the years, the report shows that risk factors for cardiovascular diseases in China are still widespread, and the number of cardiovascular diseases continues to increase [7–9]. The report analyzes the distribution of heart disease in urban and rural areas in detail and believes that cardiovascular disease is the main heart disease. Judging from the mortality rate of urban and rural residents over the years, among them, the proportion of rural areas is not large, accounting for about two-fifths, while the proportion of cities is as high as three-fifths, which is 20% higher than that of rural areas [10–13]. In addition, in terms of the number of heart disease patients, the number of people in urban and rural areas has increased. And the age is getting younger and younger. The report shows that in the next 10 years, this number will continue to rise rapidly. According to the investigation of the risk factors of heart disease, the incidence of hypertension is closely related to the prevalence of most patients in our country. In my country, the number of hypertensive patients in 2018 was 290 million, and the adult prevalence rate reached about 20%. In addition, infants and young children are also a very vulnerable group of people. The results of various investigations and studies have shown that for the development of heart disease, all walks of life are actively and effectively coping with the disease. As a serious disease, its early diagnosis is still challenging. Many people do not realize that they have heart disease. In fact, as many as 25% of heart disease patients are asymptomatic, even though their heart blood flow is insufficient. This condition is called “silent heart disease.” This leads to some complications, such as heart failure. When the heart can no longer pump enough blood, the body cannot function normally [14].

The health index of North China and East China is relatively high at about 80, the rest of the region is around 50, and the health index of Southwest China is only about 30 [15].

With the continuous development of ultrasonic diagnostic technology, color Doppler ultrasonography with high discrimination ability is widely used in the diagnosis of clinical diseases, which is of great significance for the preoperative diagnosis and evaluation of heart disease. Color Doppler ultrasound has very high clinical diagnostic value for common heart diseases such as cardiomyopathy, valvular heart disease, congenital heart disease, hypertensive heart disease, and coronary atherosclerotic heart disease, as shown in Figure 1.

The result of medical diagnosis and the predicted result are both negative and negative, that is, whether the result is a certain disease or not, once the diagnosis is incorrect or the prediction is not in place, it will be judged that it is not the cause of the disease. However, there will be a lack of relevant research for other diagnosis and treatment with the same or similar symptoms. At present, the main research approach in medicine is to use a large amount of medical data collected from a wide range of sources to conduct diagnosis and treatment research in the field [16, 17]. The diagnosis of heart disease and the field of disease prevention and treatment have the same characteristics.

Therefore, the main research focus at present is to expand more effective and accurate diagnosis models in the medical diagnosis system of heart disease, combined with the subject area of data mining algorithms. Use cardiology medical data to conduct data mining and data analysis research, and provide auxiliary medical diagnosis for reducing the error of medical diagnosis.

## 2. Related Work

In recent years, the rapid development of ultrasound imaging and Doppler technology has played an important role in the diagnosis of congenital heart disease. When diagnosing congenital heart disease with simple left-to-right shunt, it can show abnormal blood flow. Abnormal blood flow signals to determine the pathological type. According to the QP/QS estimation of the left and right ventricular shunt flow, ASD can distinguish primary and secondary pores, and PDA can distinguish the biphasic flow of the aortic blood flow to the pulmonary artery when it passes through the patent ductus arteriosus. In the diagnosis of complex congenital heart disease, pulmonary artery stenosis can show high-speed turbulence. In pulmonary hypertension, pulmonary artery expansion can prompt the identification of the pulmonary artery. Abnormal pathological changes such as coronary atrioventricular fistula, pulmonary vein odor drainage, and ultrasound color puller can track blood flow signals in abnormal channels and can display all the formations to determine the type of disease. The heart is composed of 3 segments and 2 connections. The 3 segments are the new chamber, the ventricle, and the aorta [18]. The connection between the ventricle and the aorta and the connection between the atrioventricular when the two are connected. When the position of the heart is abnormal, the positions of the atria and ventricles cannot be recognized based on the spatial position, but based on the anatomy of the heart. In the diagnosis of complex congenital heart disease, attention should be paid to the application of sequential segmentation diagnosis. For patients with simple heart disease, attention should also be paid to its use. Therefore, the doctor should have a three-dimensional space concept for the heart scan during the examination and use continuous tracking to check the conditions of the atrium, ventricle, and aorta. When diagnosing ventricular septal defect, it is necessary to adjust the sensitivity of the instrument, use the best two-dimensional image to scan the right ventricular outflow tract, and pay attention to the abnormal blood flow starting position and initial speed when checking the right ventricular outflow tract stenosis. The blood flow starts at the narrowest part of the right ventricular outflow tract, and the rate of outflow increases. When complicated congenital heart disease is combined with other heart malformations, it is necessary to gradually scan to prevent missed diagnosis and to determine the location of the intracardiac shunt-type malformation and the direction of the shunt. In short, color Doppler ultrasound imaging technology is reliable and intuitive in diagnosing congenital heart disease, can sensitively display abnormal shunts, and can provide blood flow information at the narrowest part and estimate the severity and prognosis of congenital heart disease [19].

The information in the medical data set is vague or incomplete. Under such difficult circumstances, the use of advanced learning methods such as the theoretical knowledge of data mining technology to apply this complex medical clinical data set, combining the medical field and data mining technology into one, can solve the above-mentioned problems. The combination of research in the two fields allows doctors to accurately and quickly diagnose the causes of patients and plays a vital role in studying the law of human diseases [20, 21].

For the needs of different diseases and pathologies, experts and scholars in the relevant medical diagnosis field have worked hard to develop various medical diagnosis expert systems, general systems, and special systems to assist in diagnosis and treatment. This kind of system can assist doctors in diagnosis by inputting corresponding information in the diagnosis system through analysis and calculation of big data, etc., which can provide doctors and patients with auxiliary reference and give preliminary diagnosis and treatment suggestions. The clinical experience and rich medical knowledge can be saved in the auxiliary diagnosis system, which can not only provide auxiliary reference for less experienced doctors to reduce the probability of misdiagnosis but also make preliminary diagnosis. As a combination of data mining and medical field, the medical assistant diagnosis and treatment system has obtained many research results at home and abroad [22–24]. At the same time, the algorithm model of support vector machine (SVM) is established, and the classification accuracy has been greatly improved. At present, financial, environmental, industrial, and other industries in various fields have more applications of the results of data mining technology, which all promote the development of data mining technology [25–27]. Combining data mining technology with the medical diagnosis system of heart disease is the main research content of this article [28]. According to the classic algorithm in data mining technology, the theoretical study is carried out, and the selected classification algorithm is used to analyze the heart disease data set obtained from the UCI machine learning database [29]. Carry out analysis and research and build a classifier. Compare and analyze the performance of different classifiers and optimize them.

## 3. Method

### 3.1. Ultrasound Diagnosis Method

The detection instrument is a GE VIVID3 color Doppler ultrasonic diagnostic instrument, which uses new ultrasonic diagnostic technology to report the patient's heart structure and heart blood flow distribution. Comprehensive examination of the patient's apex, subxiphoid, suprasternal fossa, parasternal, and other acoustic windows, segmented diagnosis according to the sequence of congenital heart disease, the heart is divided into three segments of atrium, ventricle, and aorta for examination one by one, using two-dimensional and M-mode echocardiography measures and observes and records the inner diameter of each atrium, ventricle, and large blood vessels, valve and ventricular wall thickness, and amplitude of motion. Measure left ventricular end-diastolic volume and end-diastolic volume index. The ejection fraction was measured using the Simpson method. Calculate the ratio of the pulmonary circulation to the systemic circulation, the blood flow distribution of the heart and large vessels, measure the starting position and width of the abnormal blood flow and the flow velocity, keep the sampled volume and blood flow direction as parallel as possible, observe and record the abnormal blood flow nature, direction, speed, and time phase.

### 3.2. Data Mining Implementation Method

In 1989, at the 11th International Joint Artificial Intelligence Conference, the term Knowledge Discovery in Database (KDD) was first proposed. In the following three years, three special conferences were held on it. Experts and scholars in various fields and program application development scholars have conducted intensive discussions on data processing, information acquisition, and other issues. There are many international conferences in the field of data mining. After decades of hard work, data mining technology has achieved rapid development in all aspects and fields of research and has yielded fruitful results. Many data mining software products have been developed and listed by various software companies and have been widely used in Europe, North America, and other countries. Agrawal and others have developed two patents when they were at IBM, both of which are related to association rules in data mining. Subsequently, SAS and other companies developed a data mining system integrating many mature technologies.

**Step 1 (business understanding).**

There are many misunderstandings about business understanding. The essence of business understanding is to first determine the data mining problems to be implemented and the desired goals. The general process is to first conduct business research and understanding, clarify the positioning of the problem, formulate corresponding goals, and finally conduct business analysis. Only a comprehensive understanding of business methods can be implemented accurately and effectively.

**Step 2 .**

The indicator design is based on the premise of step 1; after sorting out and understanding the problem, find a suitable analysis method as a theoretical support to know the indicator design of the model to ensure the comprehensiveness of the indicator system.

**Step 3 (data extraction).**

Data extraction ensures the integrity, availability, and completeness of the modeled data. Data extraction: extract the data needed for modeling. Data cleaning: data cleaning is to deal with data loss, redundancy, and other issues. Data audit: data audit is an audit of data statistics, data sources, and data statistics. Data integration: data mining wide table construction.

**Step 4 (data exploration).**

The exploration of data involves two aspects. The first is to detect, analyze, and verify the original data. Ensure that it meets the original intention of the indicator design and the business meaning; secondly, according to the needs of building the model, part of the data source processing, standardization processing, discretization processing, etc., so that different indicator attributes are mathematically calculated on the same scale and evaluation.

Data standardization (standardization) processing is a key step in the preprocessing steps of the initial data set, and it is also a basic work in data mining technology. The evaluation of different attributes and different indicators of the data set usually affects the dimensionality of the data, which will affect the results of data analysis. In order to eliminate the dimensional influence between indicators (features), it is necessary to use the method of data standardization that the original data set can have the same division indicators. After using the data standardization method, the data set can be uniformly divided into the same quantitative level interval. This is suitable for subsequent comprehensive comparative evaluation.

1. Min–max normalization

(1) $$\begin{array}{c} Y=\frac{X-X_{\min}}{X\min_{\max}*\left({X\text{minmin}}_{\max}\right)}. \end{array}$$

(2) Zero mean normalization

(2) $$\begin{array}{c} Y=\frac{X-\mu }{\sigma }. \end{array}$$

(3) Fuzzy quantification and standardization

(3) $$\begin{array}{c} Y=\frac{1}{2}+\frac{1}{2}*\sin\left[\frac{\pi }{X_{\max}-X_{\min}}*\left(X-\frac{X_{\max}-X_{\min}}{2}\right)\right]. \end{array}$$

Discretization is generally a technical method commonly used in programming, which can effectively reduce time complexity. The basic idea is to consider only the values that need to be used in many possible situations. Discretization of data can improve inefficient algorithms or even implement an algorithm that is impossible to achieve. To master this idea, one must understand the characteristics of this method from a broad perspective. When processing some massive data sets, they cannot be used as array subscripts to save the corresponding attributes. If there are independent interattribute relationships between these data attributes, the data can be discretized for this batch of data sets. When the data set depends only on the relative attribute size of the data and not on the size of the data, the data can be discretized.

**Step 5 .**

Algorithm selection.

**Step 6 (model evaluation).**

There are many aspects to evaluate the evaluation criteria of model evaluation, and the evaluation methods and tools are also different.

**Step 7 (model release).**

This step focuses on providing end-to-end theme solutions to business problems, improving the effectiveness and value of data mining applications; it is a set of end-to-end and complete data mining theme solutions, rather than simple data mining results.

**Step 8 (model optimization).**

Perform corresponding tests and evaluations on the released models, and do a good job of timely optimization and timely processing of model algorithms.

### 3.3. Source and Processing of Clinical Care of Heart Disease

Experiment in numerous classification algorithms: comparing these experimental results, the highest correct classification rate is obtained as the best model for diagnosing heart disease, which is used in the heart disease medical auxiliary diagnosis system to provide a predictive auxiliary system for the timely prevention of heart disease. The paper is based on the UCI database of the University of California Irvine. Most of the UCI databases are data sets for machine learning research and analysis, which are used for data mining algorithms and machine learning commonly used data sets. The clinical data set is the research object, in which the conditional attributes are multiple factors that may lead to heart disease, and the decision-making attributes are the final diagnosis results. There are 13 test attributes in total. The category attributes are category A, which means there is no heart disease, and category B, which means there is heart disease. There are a total of 270 samples.

From the above table, for example, in this article, gender (male, female) is represented as 0, 1, respectively. In this way, all the discretized data sets needed in this article are generated. In the paper, the data sample points of the medical data set are uniformly divided into two parts, the test set and the training set: (1) age, (2) sex, (3) chest pain type, (4) resting blood pressure, (5) serum cholesterol, (6) fasting blood sugar content, (7) resting electrocardiographic result, (8) maximum heart rate, (9) exercise-induced angina, (10) the old peak-ST motion is relative to the stress induced by other motions, (11) the slope of the peak exercise ST segment, (12) the number of major vessels colored by fluoroscopy, and (13) thalassemia.

The final classification attribute class of the data sample set is A, B. A represents the presence of heart disease, and B represents the absence of heart disease.

Standardized attributes: in order to make the model in the experiment process better, the determined value of each attribute will be used to divide the characteristics of its own attributes. The purpose of this is to achieve between each attribute. The discretized value between 0 and 1 strengthens the training of the model and provides the best experimental results.

### 3.4. Experimental Data Preprocessing

Open the data set data.csv file with Weka software, and save it as a data file. Make it saved as Weka software's own data format type. Arff file, it automatically becomes a histogram of each attribute.

The medical attributes of the medical clinical data set are tested for attribute correlation. Determine the degree of correlation of each attribute, and determine the correlation. The attributes are deleted. Use the Gain Ratio Attribute in the Attribute Evaluator under the Select attribute column of the Weka software and the Ranker in the Search Method to check the correlation of sample attributes.

Therefore, it can be obtained that the correlation degrees of the three sample attributes of attribute 4, attribute 5, and attribute 6 are all zero. Due to the different data types among the various attributes of the medical clinical data set, it is convenient for data processing and data type classification. Now, the data set is processed for discretization and normalization of data to support subsequent data modeling.

### 3.5. Data Mining Algorithm

Data mining algorithms refer to a series of mathematical formulas or codes used in the establishment of key models. Algorithms are prepared for analyzing data and creating models. Before modeling, first analyze the given data and use different algorithms to model and analyze it. You can also use predictive algorithms to analyze the future based on the established model, time period for predictive analysis. Among the data mining algorithms, the ten most classic algorithms include *K*-means algorithm, support vector machine (SVM for short), maximum expectation algorithm (EM for short), C4.5 algorithm, Page Rank, Ada Boost, *K* nearest neighbor classification algorithm (KNN), naive Bayes model (NBC), association rule frequent itemset algorithm (Apriori algorithm), and classification and regression tree (CART). Of course, more and more scholars have improved these algorithms, and the accuracy of data mining has been greatly improved.

Decision tree is a method of approximating discrete function values, and it is also a commonly used classification algorithm for classic data mining. The earliest origin was in the 70s of the last century. Its core theory is to carry out an effective classification process for a series of data sets, and the final classification result shows the shape of a tree like the shape of a tree.

The most commonly used decision trees are decision tree ID3 algorithm, decision tree C4.5 algorithm, and decision tree CART algorithm. This article mainly uses the decision tree C4.5 algorithm.

The decision tree C4.5 algorithm can be used for classification problems and also for regression problems. Algorithm C4.5 is not directly used for information gain. At the same time, it has made great optimizations in terms of predictive variable pruning technology, derivation rules, and lack of value processing. Compared with other decision tree algorithms. It uses information, information gain rate, etc. to select the best classification.

1. Information entropy Ent(*S*)

(4) $$\begin{array}{c} \text{Ent}\left(S\right)=-\overset{k}{\underset{i=1}{\sum }}P\left(C_{i},S\right)\log_{2}\left(P\left(C_{i},S\right)\right). \end{array}$$

(2) Information entropy Ent(*A*, *T*; *S*)

(5) $$\begin{array}{c} \text{Ent}\left(A,T;S\right)=\frac{\left|S_{1}\right|}{\left|S\right|}\text{Ent}\left(S_{1}\right)+\frac{\left|S_{2}\right|}{\left|S\right|}\text{Ent}\left(S_{2}\right). \end{array}$$

Information Gains(*A*, *T*; *S*)

(6) $$\begin{array}{c} \text{Gains}\left(A,T;S\right)=\text{Ent}\left(S\right)-\text{Ent}\left(A,T;S\right). \end{array}$$

The characteristics and advantages of the decision tree C4.5 algorithm are easy to understand, as well as the interpretation and analysis of the results. There is no high computational complexity, and the foundation is not high. The knowledge level can generally understand the meaning displayed by the decision tree; at the same time, it can be used in the data set. There are many attributes for constructing a decision tree, and it can process big data in a relatively short time that is feasible and has good classification results; it can also process data sets of different data types and subtype attributes at the same time, and missing data can also be handled. However, there is also a disadvantage that the results of information gain will be biased in data sets with different categories, and overfitting will occur. At the same time, being very sensitive to noise data will become a problem when modeling and processing data.

The artificial neural network (ANN) development environment is based on a very complex biological neural network. The human brain is composed of thousands of highly interconnected neurons, and each neuron has hundreds of connections. Artificial neural network uses methods such as imitating biological neurons and using mathematical expressions to successfully introduce this concept. Neural network algorithms are a kind of supervised learning. In the research of neural network algorithms, the basic unit neuron is the basis of the research, and the general neuron model is in the form of multiple input information and one output source, as shown in Figure 2.

*X*_1_, *X*_2_, ⋯, *X*_*n*_ means the input data set; *a* is the output variable of the neuron model; *W*_1_, *W*_2_, *W*_3_, ⋯, *W*_*n*_ is the intensity of action in the neuron model; *Σ* is the data information feedback; *b* is the adjustment threshold; *σ* is the characteristic function of neuron activity.

(7) $$\begin{array}{c} X_{i}=\sum W_{j}X_{j},\\ a=F\left(X_{i}^{\prime }\right)=F\left(\sum w_{j}x_{j}-\sigma \right). \end{array}$$

After appropriate adjustments are made to the comprehensive input *X*_*i*_, it is necessary to further describe this relationship with a characteristic function to generate a new output *a*.

The advantage of the neural network algorithm is that it has strong fault tolerance to noise nerves and can fully have associative memory capabilities and very close to complex nonlinear relationships; parallel distributed storage capabilities and learning capabilities are extremely strong; at the same time, distributed processing ability also has obvious advantages over other algorithms. The disadvantage is that the learning time is too long and the modeling time is relatively long; and it requires a large number of parameter settings and the inability to intuitively observe the learning process, which makes the results difficult to interpret and affects the credibility of the results.

Data mining technology is an important aspect of machine learning based on data. Starting from sample data, looking for patterns in data is a very traditional way. In the applied research of statistics, theories based on the laws of machine learning are gradually emerging. The support vector machine algorithm (SVM) is a data mining algorithm based on statistical learning theory and was jointly proposed by Boser and others in 1992.

The basic idea of the support vector machine algorithm (SVM): the black dot and the white dot under the condition of linear separability represent two types of samples, the *H* line is the classification line between them, and line *H*_1_ is the line connecting the positions of all white sample points and the *H* line, the closest straight line; line *H*_2_ is the sample point where the black points of all samples are closest to the classification surface. The straight line *H*_1_ and the straight line *H*_2_ are the two parallel and shortest straight lines parallel to the classification straight line *H*, between the straight line *H*_1_ and the straight line *H*_2_. The distance is the classification interval.

Cobweb is translated as spider web model or spider web theory, which is an economic model that can explain why prices may be affected by cyclical fluctuations in certain types of markets. It describes the cyclical supply and demand in the market, where the output must be selected before the price is observed. The producer's expectation of prices is based on observations of previous prices. Nicholas Kaldor analyzed the model in 1934 and coined the term “cobweb theorem.” With the rise of the Internet of Things and data mining technology, the cobweb algorithm is defined as a model-based method. This model method assumes a model for each attribute in the data set, the object is on each node and calculates the result of the calculation. The location where the highest classification utility is generated should be a good choice for the object node. However, if it does not belong to any existing concept in the tree, instead create a new class for the object.

The advantage of the cobweb algorithm is that the algorithm does not require human intervention and set the number of clustering parameters. It automatically corrects and divides the data set, which reduces manual participation and makes the results of later classification using SVM more accurate. This paper is based on the combination of cobweb clustering algorithm and support vector machine classification algorithm; now the data set is used for model clustering method so that it can be clustered on a large scale, and the similarities are clustered into one category, and then, the support vector machine is used for classification. Algorithm for classification research, the use of Co-SVM has greatly improved the accuracy of classification compared with decision trees, neural networks, and support vector machines. Through rigorous experimental analysis and research, the clustering results obtained by the cobweb clustering algorithm are applied to the SVM algorithm for classification and analysis. The data mining algorithm has a strong generalization ability and at the same time solves the problem of the difficulty of dividing the high-dimensional space of the SVM algorithm.

## 4. Experiment and Result

The essence of the heart disease medical diagnosis system is to output the binary classification result of yes or no. Analyze the most important accuracy results first, and then, compare and analyze the prediction result graph, ROC curve, and modeling time. The prediction accuracy and precision of the algorithm are very significant, as shown in Figures 3 and 4.

The result cluster map is the final classification prediction result map of the Co-SVM algorithm. It can be seen from the figure that the small squares are the wrong predictions, and the prediction accuracy and precision of the algorithm are very significant.

In medical research, the diagnostic model of the evaluation system is generally based on the ROC curve, which also displays the abstract prediction data more vividly and concretely. The evaluation basis of the ROC curve is based on the curve being close to the upper left of the marked axis as the reference basis. According to the evaluation results of the four algorithms, the Co-SVM algorithm performs better than the decision tree, neural network, and SVM algorithm, as shown in Figure 5.

After passing the evaluation method mentioned in Chapter 2, with the help of 10-fold cross-validation, the four models will be compared and analyzed in three aspects: Kappa statistics, root square error, and relative absolute error. The Kappa coefficient is used to judge the difference between the classification results of the classifier and the random classification. It is a consistency test. Kappa is the decimal in the area [−1, 1]. When the classification effect of the model classifier is poor, the statistic is close to -1; when the effect of the model classifier is the same as the effect of random classification, the statistic is 0, that is, the model classifier does not play any role; the model classifier has a different result compared with the random classification. And the classification effect is better, the statistic is 1. The result of the statistics is positively correlated with the evaluation index of the model classifier and the corresponding accuracy rate. Therefore, the larger the value of the statistic, the better the classification effect and classification performance of the model classifier. The results of root square error and relative absolute error are negatively correlated with the accuracy of the classifier, that is, the smaller the value, the better the effect of the classifier, as shown in Figure 6.

The Kappa statistic of the Co-SVM algorithm is 0.723, which is 16.9%, 23.9%, and 3.4% higher than the Kappa statistic of the other three algorithms, respectively. Comparing the other two, the root mean square error and average absolute error of the Co-SVM algorithm are, respectively, 9.38% and 23.42% lower than the decision tree algorithm and 17.17% and 14.37% lower than the neural network algorithm. It is 4.13% and O.H% lower than the support vector machine algorithm. In summary, after the analysis of the error results, the Co-SVM algorithm has the lowest error, and the effect of classification is better, as shown in Figure 7.

The time-consuming analysis is through WEKA's algorithm modeling and analysis. In the modeling time analysis, the Co-SVM algorithm is 0.015, and the support vector machine is 0.015, which is 0.525 and 0.025 less than the BP neural network algorithm and the decision tree, respectively. Therefore, the form of the support vector machine during the time analysis of the heart disease data set is compared with the BP algorithms and decision tree modeling is realized more quickly and efficiently.

In summary, with the help of the above decision tree C4.5 algorithm, BP neural network algorithm, support vector machine algorithm, and Co-SVM algorithm, four types of classifiers have been carried out in the four aspects of accuracy, ROC curve, error analysis, and modeling time. Through comparative evaluation, it is clear that the classifier constructed by the Co-SVM algorithm exhibits the best operational performance during the establishment of the corresponding heart disease diagnosis classification model for the heart disease data set.

In addition, the research in this article found that one of the main causes of death due to heart disease is not aware of it in the early stage of disease development. Regular physical examination can help to detect the disease in the early stage. If heart disease can be detected in time, it can be properly treated. Smoking, unhealthy diet, and irregular exercise can all induce heart disease, which also requires individuals to adjust their habits to avoid the occurrence and development of the disease.

## 5. Conclusion

Through the understanding of various aspects, there are many researches on heart disease based on data mining algorithms, mainly focusing on the application of neural network algorithms and the application of support vector machine algorithm kernel functions. In this paper, four data mining algorithms, including decision tree C4.5 algorithm, BP neural network algorithm, support vector machine algorithm, and Co-SVM algorithm, are selected to establish a heart disease diagnosis classifier.

The thesis conducts research on the diagnosis of heart disease and conducts research and comparative analysis on the four algorithm diagnosis models of decision tree C4.5 algorithm, neural network algorithm, support vector machine algorithm, and Co-SVM algorithm. Based on the heart disease clinical data set in the UCI database specifically for machine learning research as the research object, the decision tree C4.5 algorithm, neural network algorithm, support vector machine algorithm, and Co-SVM algorithm are used to establish heart disease diagnosis. The classifier, through experimental comparison and analysis, selects the best classification algorithm Co-SVM algorithm based on the comparison of the obtained results. The experimental results show that the proposed Co-SVM algorithm has a higher accuracy rate than the other three classic algorithms, and the effectiveness of the Co-SVM algorithm is verified by the evaluation results of multiple algorithms. By applying the Co-SVM algorithm in the medical diagnosis system, it helps to assist doctors in making more accurate and precise diagnosis of the condition [30].

At the same time, the application of color Doppler ultrasound with high discriminative ability to diagnose clinical diseases is of great significance for the preoperative diagnosis and evaluation of heart disease. Color Doppler ultrasound has high clinical diagnostic value for common heart diseases such as cardiomyopathy, valvular heart disease, congenital heart disease, hypertensive heart disease, and coronary atherosclerotic heart disease.

## Figures and Tables

**Figure 1:** National heart health index.

**Figure 2:** Model.

**Figure 3:** The accuracy of the four algorithms.

**Figure 4:** The recall rate of the four algorithms.

**Figure 5:** ROC curve comparison chart.

**Figure 6:** The errors of the four algorithms.

**Figure 7:** The time of the four algorithms.

## Data Availability

The datasets used and analyzed during the current study are available from the corresponding author upon reasonable request.
